The article "Clinical Efficacy of Xueshuantong plus Urokinase in the Treatment of Sudden Deafness" was retracted in 2023. Reasons: unreliable results or conclusions; concerns about the data; concerns about the peer review; concerns about the citations.

# Clinical Efficacy of Xueshuantong plus Urokinase in the Treatment of Sudden Deafness

**DOI:** 10.1155/2022/7775556

**Published:** 2022-06-29

**Authors:** Yanling Wang, Jian Wang, Xiulan Chen

**Affiliations:** ^1^South China Hospital affiliated to Shenzhen University, The ENT Department, Shenzhen 518100, China; ^2^The ENT Department, Qinghai Provincial People's Hospital, Xining, Qinghai 810007, China

## Abstract

**Objective:**

To investigate the clinical effect of Xueshuantong combined with urokinase in the treatment of sudden deafness.

**Methods:**

A total of 90 patients with sudden deafness who were treated in South China Hospital affiliated to Shenzhen University from June 2019 to August 2020 were recruited and assigned (1 : 1) into the control group (*n* = 45, urokinase) and the experimental group (*n* = 45, Xueshuantong plus urokinase) according to the different treatment methods. The clinical treatment effect, the degree of tinnitus, the average auditory valve of the damaged frequency, and the changes in hemorheology (plasma viscosity, whole blood high-shear reduced viscosity, whole blood low-shear reduced viscosity, hematocrit, and fibrinogen) were compared between the two groups of patients.

**Results:**

The treatment with urokinase and Xueshuangtong injection in the experimental group resulted in a significantly higher clinical treatment effect when compared with the treatment in the control group (*P* < 0.05). After treatment, the degree of tinnitus and the average auditory valve of the damaged frequency in the experimental group were significantly lower than those in the control group (*P* < 0.05). The levels of hemorheology (plasma viscosity, whole blood high-shear reduced viscosity, whole blood low-shear reduced viscosity, hematocrit, and fibrinogen) in the experimental group after treatment were significantly lower than those in the control group (*P* < 0.05).

**Conclusion:**

The clinical effect of Xueshuantong combined with urokinase in the treatment of patients with sudden deafness is remarkable, and it can effectively improve the hearing level and hemorheology-related indexes of patients, and it thus merits clinical application.

## 1. Introduction

Sudden deafness is one of the common diseases of otolaryngology, and it falls into the category of sudden sensorineural hearing loss [1]. The main manifestations of the disease are deafness, tinnitus, earplugs, nausea, and dizziness [2], greatly compromising the patient's daily life [3]. Though clinical cause of the disease is still unclear, several contributors such as virus infection theory, circulatory disorder theory, and immune theory have been identified [4]. At present, clinical-related research believes that the pathogenesis of sudden deafness is mainly related to viral infection, blood circulation disorder, eardrum labyrinth rupture, and autoimmune function, among which the theory of ear microcirculation has been widely recognized by the academic community [5]. The blood of the inner ear mainly comes from the labyrinthine artery of the human body. Since this artery has no collateral circulation, once thrombosis or vasospasm occurs, it would lead to ischemia, hypoxia, and microcirculation disturbance in the patient's ear, which further damages the inner ear and even causes irreversible deafness [6]. A large number of clinical studies have shown that vascular disease plays a very important role in sudden deafness, and systemic dysfunctions such as coagulation and fibrinolysis in the labyrinthine arteries often contribute a lot to sudden deafness [7]. Therefore, improving the inner ear microcirculation of patients is of great significance to minimize the possibility of sudden deafness [8].

The article "Clinical Efficacy of Xueshuantong plus Urokinase in the Treatment of Sudden Deafness" was retracted in 2023. Reasons: unreliable results or conclusions; concerns about the data; concerns about the peer review; concerns about the citations.

Urokinase is one of the commonly used drugs for the clinical treatment of patients with sudden deafness [9]. As a thrombolytic drug, it can act well on the endogenous fibrinolytic system and catalyze the cleavage of plasminogen into plasmin. It not only degrades protein clots but also degrades fibrinogen, coagulation factor V, and coagulation factor VIII in the blood circulation, thereby playing a role in thrombolysis [6]. However, relevant clinical studies have pointed out that the therapeutic effect of urokinase alone in the treatment of sudden deafness is not ideal [10].

According to the theory of traditional Chinese medicine, sudden deafness is related to qi stagnation, blood stasis, and vein obstruction, which is consistent with the viewpoint of sudden deafness caused by the blocked inner ear blood supply in modern medical theory [11]. Based on this, the combination of traditional Chinese medicine for promoting blood circulation and dredging collaterals can be considered in clinical treatment of this disease [12]. Xueshuantong injection has the effect of rapidly dissolving thrombus and improving the blood supply of the patient's body. It can effectively reduce the pathological damage caused by ischemia, thereby improving the blood microcirculation of the inner ear [13]. At present, there is a paucity of evidence on the effect of Xueshuantong combined with urokinase in the treatment of patients with sudden deafness. The purpose of this study was to explore the clinical effect of Xueshuantong combined with urokinase in the treatment of sudden deafness.

## 2. Materials and Methods

### 2.1. Study Population

A total of 90 patients with sudden deafness who were treated in South China Hospital affiliated to Shenzhen University from June 2019 to August 2020 were recruited and assigned (1 : 1) into the control group (*n* = 45) and the experimental group (*n* = 45) according to the different treatment methods. The patients were informed about the study and signed the informed consent voluntarily.

The article "Clinical Efficacy of Xueshuantong plus Urokinase in the Treatment of Sudden Deafness" was retracted in 2023. Reasons: unreliable results or conclusions; concerns about the data; concerns about the peer review; concerns about the citations.

### 2.2. Inclusion and Exclusion Criteria

The inclusion criteria were as follows: (1) the clinical diagnostic criteria for sudden deafness were met; (2) age 18∼70 years old. The exclusion criteria were as follows: (1) patients with cardiovascular and cerebrovascular diseases and bleeding diseases; (2) patients with poorly controlled hypertension or diabetes; (3) those who had taken anticoagulant drugs within 1 month before enrollment (4) pregnant and lactating women; (5) patients with severe liver and kidney insufficiency; and (6) patients with poor compliance who could not cooperate with this study.

### 2.3. Methods

Patients in the control group were treated with 200,000 IU urokinase (manufacturer: Guangzhou Putian Chemical Pharmaceutical Co., Ltd.; approval number: H44024035) [9] with 100 ml of normal saline, via intravenous infusion within 30 minutes, once a day. On the basis of the treatment in the control group, the patients in the experimental group were given 450 mg Xueshuantong injection (manufacturer: Guangxi Wuzhou Pharmaceutical Group Co., Ltd.; approval number: Z20025652) with 500 ml of 5% glucose injection via an intravenous drip, 1 time/d. Both groups were treated for 1 month.

### 2.4. Outcomes

1. Clinical treatment efficiency: cured: the average hearing valve of the damaged frequency returns to the normal level; markedly effective: the average hearing valve of the damaged frequency is increased to more than 30 dB; improved: the average hearing valve of the damaged frequency is increased to 15–30 dB; ineffective: the condition does not meet the above standards or even aggravates. Total effective rate = (cured + markedly effective + improved)/total number of cases × 100%.
2. Determination of the degree of tinnitus and the average auditory valve of the damaged frequency: according to the tinnitus environment, tinnitus duration, tinnitus impact on sleep, tinnitus impact on life and work, tinnitus impact on mood, and the overall feeling of patients with tinnitus, the score is 0∼3 from light to severe. The higher the score, the more serious the damage.
3. Hemorheology: 5 ml of fasting venous blood was drawn from patients before and after treatment, lithium heparin was used for anticoagulation, and an automatic hemorheology detector was used to detect the plasma viscosity, whole blood high-shear reduced viscosity, whole blood low-shear reduced viscosity, hematocrit, and fibrinogen index levels.

The article "Clinical Efficacy of Xueshuantong plus Urokinase in the Treatment of Sudden Deafness" was retracted in 2023. Reasons: unreliable results or conclusions; concerns about the data; concerns about the peer review; concerns about the citations.

### 2.5. Statistical Analysis

The data analysis was performed using software SPSS20.0, measurement data are expressed as ($\bar{x}\pm s$), and the independent samples *t*-test was used for comparison; enumeration data are expressed as the number of cases (rate), and the chi-square test was used for comparison. Statistical significance was set at *P* < 0.05.

## 3. Results

### 3.1. General Data

The control group included 24 males and 21 females, the mean age was (52.57 ± 6.58) years, the mean disease duration was (3.79 ± 2.87) days, and 28 patients were unilateral and 17 bilateral. The experimental group included 25 males and 20 females, the average age was (52.72 ± 6.63) years, the average disease duration was (3.75 ± 2.91) days, and 26 cases were unilateral and 19 bilateral. There was no significant difference in baseline data between the two groups of patients, as shown in Table 1.

### 3.2. Clinical Treatment Effects

In the control group, there were 11 cases of cured, 16 cases of markedly effective, 9 cases of improved, and 9 cases of ineffective, with a total effective rate of 80% (36/45). In the experimental group, there were 27 cases of cured, 10 cases of markedly effective, 7 cases of improved, and 1 case of ineffective, with a total effective rate of 98% (44/45). The treatment with urokinase and Xueshuangtong injection in the experimental group resulted in a significantly higher clinical treatment effect when compared with the treatment in the control group (*P* < 0.05, Table 2). In addition, no significant adverse reactions were observed in either study group.

### 3.3. Tinnitus Degree and Damaged Frequency Average Listening Valve

Before treatment, the degree of tinnitus and the average auditory valve of the damaged frequency were comparable (all *P* > 0.05). After treatment, the above indicators were all decreased, and the much lower results were observed in the experimental group (*P* < 0.05), as shown in Table 3.

### 3.4. Hemorheology Indexes

The levels of hemorheology (plasma viscosity, whole blood high-shear reduced viscosity, whole blood low-shear reduced viscosity, hematocrit, and fibrinogen) were comparable between the two groups. After treatment, the above indicators were all decreased and lower in the experimental group (*P* < 0.05, Table 4).

## 4. Discussion

The results showed that the degree of tinnitus and the average auditory valve of the damaged frequency in the two groups were improved after treatment, which indicates that urokinase thrombolysis can relieve the symptoms of patients and is effective to improve the hearing of patients [14]. Urokinase is a commonly used thrombolytic drug in clinical practice and plays a role in thrombolysis [15]. However, the effective dose of thrombolytic drugs presents individual differences, so it is challenging to accurately manage the dose in clinical practice, which results in poor efficacy in most cases. Possibly, the degradation of fibrinogen would lead to hyperfibrinolysis in the whole body, thus resulting in the digestive tract hemorrhage, cerebral hemorrhage, and other side effects [16]. According to the theory of TCM, sudden deafness is associated with the stagnation of qi and blood in the body and the obstruction of blood vessels. Armed with this knowledge, the combination of traditional Chinese medicine for promoting blood circulation and dredging collaterals might be a feasible strategy in clinical treatment of this disease [17]. According to the theory of TCM, it can significantly mitigate the symptoms of sudden deafness. Studies have confirmed that acupuncture points such as the Yifeng point contribute to enriching yin and purge fire so as to effectively promote the body ErCong intruders. Xueshuantong injection is made from the extract of traditional Chinese medicine, that is, Panax notoginseng. Its main active ingredient, Panax notoginseng saponins, can favorably promote blood circulation and remove blood stasis and has functions of antithrombotic and antiplatelet aggregation [18]. The findings of the present study showed that the clinical treatment effect of the patients in the experimental group was significantly superior to that in the control group, suggesting that Xueshuantong combined with urokinase produces a remarkable efficiency in the treatment of patients with sudden deafness. The possible explanation may be that the total saponins of Panax notoginseng in Xueshuantong can inhibit thrombin-induced platelet aggregation, thus inhibiting the formation of thrombus in the body. Also, it can scavenge oxygen free radicals, thereby inhibiting lipid peroxidation and alleviating the damage of ischemia-reperfusion in the body. All these reduce the damage to tissue and organ function caused by ischemia [19]. To the best of our knowledge, Xueshuantong in the treatment of deep vein thrombosis of the lower extremities could significantly reduce the blood viscosity of the patient [20]. Notably, we also compared the hemorheological indicators of the patients and found that Xueshuantong can effectively improve the hemorheological indexes of patients, which further consolidates its feasibility on thrombosis [21]. In this study, the Xueshuantong capsule has good safety, but the safety of long-term applications still needs investigation. However, there were still some limitations in this study. First, the long-term clinical outcomes were not assessed. Second, the blind method was not used in the study, which might result in bias due to subject and investigator factors. Third, the number of patients included in this study was small, which might compromise its generalization. In the future, randomized controlled studies with a large sample size and long follow-up are needed.

The article "Clinical Efficacy of Xueshuantong plus Urokinase in the Treatment of Sudden Deafness" was retracted in 2023. Reasons: unreliable results or conclusions; concerns about the data; concerns about the peer review; concerns about the citations.

## 5. Conclusion

The clinical effect of Xueshuantong combined with urokinase in the treatment of patients with sudden deafness is remarkable, and its treatment method can effectively improve the hearing level and hemorheology-related indexes of patients, and it merits clinical application.

## Figures and Tables

**Table 1:** Comparison of general data.

	Control group (*n* = 45)	Experimental group (*n* = 45)	*t*/*χ*^2^	*P*
Gender			0.164	0.685
Male	24	25		
Female	21	20		
Age (years)	52.57 ± 6.58	52.72 ± 6.63	0.157	0.876
Disease duration (d)	3.79 ± 2.87	3.75 ± 2.91	0.325	0.746
Affected ear			0.161	0.688
Unilateral	28	26		
Bilateral	17	19		

**Table 2:** Comparison of clinical treatment effects (*n*, (%)).

Groups	*n*	Cured	Markedly effective	Improved	Ineffective	Total
Control group	45	11	16	9	9	36 (80%)
Experimental group	45	27	10	7	1	44 (98%)
*χ* ^2^	—					8.274
*P*	—					0.004

**Table 3:** Comparison of the tinnitus degree and average hearing valve of damaged frequency ($\bar{\text{x}}\pm s$).

Groups	*n*	Degree of tinnitus (point)		Damaged frequency average hearing valve (dBHL)	
		Before	After	Before	After
Control group	45	12.59 ± 2.71	9.75 ± 2.14	62.11 ± 17.87	44.29 ± 16.85
Experimental group	45	12.63 ± 2.68	6.78 ± 2.03	62.09 ± 17.91	11.83 ± 14.12
*T*	—	0.094	7.377	0.091	11.465
*P*	—	0.925	<0.05	0.928	<0.05

**Table 4:** Comparison of the hemorheology indexes ($\bar{\text{x}}\pm s$).

Groups	*n*	Plasma concentration (mPa·s)		Whole blood high-shear reduced viscosity (mPa·s)		Whole blood low-shear reduced viscosity (mPa·s)	
		Before	After	Before	After	Before	After

Control group	45	2.53 ± 0.42	1.95 ± 0.30	5.52 ± 0.72	4.85 ± 0.57	14.12 ± 2.16	12.09 ± 1.41
Experimental group	45	2.50 ± 0.41	1.36 ± 0.22	5.49 ± 0.49	3.72 ± 0.51	14.07 ± 2.11	9.27 ± 1.16
*T*	—	0.693	12.764	0.397	11.150	0.103	12.636
*P*	—	0.490	<0.05	0.692	<0.05	0.918	<0.05

Groups	*n*	Hematocrit (mPa·s)			Fibrinogen (g/L)		
		Before	After		Before	After	
Control group	45	51.33 ± 3.78	47.12 ± 3.64		4.51 ± 0.65	3.57 ± 0.52	
Experimental group	45	51.29 ± 3.81	42.03 ± 3.12		4.49 ± 0.72	2.33 ± 0.34	
*T*	—	0.518	7.211		0.084	15.224	
*P*	—	0.605	<0.05		0.933	<0.05	

## Data Availability

No data were used to support this study.
